This article has been retracted.

# Systematic Evaluation of the Efficacy of Acupuncture Associated with Physical and Mental Intervention when Treating Idiopathic Tinnitus and the Improvement of Tinnitus Symptoms

**DOI:** 10.1155/2022/6764909

**Published:** 2022-08-30

**Authors:** Yan Li, Di Sang, Zeting Wu, Xuemei Cao

**Affiliations:** Acupuncture & Moxibustion Dept., The Fourth Clinical Medical College of Guangzhou University of Traditional Chinese Medicine, Shenzhen 518000 Guangdong, China

## Abstract

**Objective:**

To systematically evaluate the efficacy of acupuncture associated with physical and mental intervention when treating idiopathic tinnitus and the improvement of tinnitus symptoms, so as to supply evidence-based medicine for its popularization and adoption.

**Methods:**

PubMed, EMBASE, ScienceDirect, Cochrane Library, China knowledge Network Database (CNKI), China VIP Database, Wanfang Database, and China Biomedical Literature Database (CBM) online database were searched for the controlled trial of acupuncture associated with physical and mental intervention when treating idiopathic tinnitus. The retrieval time limit is from January 2010 to March 2022. Separately, two researchers extracted the data, and according to the Cochrane Handbook 5.3, the bias risk of each piece of literature was assessed. The collected data were measured using RevMan5.3 statistical software.

**Results:**

Finally, 5 CT articles were included in this study, with a total sample size of 282. Meta-analysis showed that the effective rate of the study group was significantly higher than that of the control group (*P* < 0.05). The scores of tinnitus disorder scale (THI) after treatment were analyzed by Meta. The THI scores of the study group after treatment were significantly lower than those before treatment. Meta-analysis of the severity of tinnitus after treatment showed that the severity of tinnitus in the observation group after treatment was significantly lower than that before treatment. There is a certain publication deviation in the literature, which may be related to the heterogeneity of the research and the small number of literatures.

**Conclusion:**

On the basis of acupuncture treatment, associated with physical and mental intervention is helpful to the recovery of patients with idiopathic tinnitus, can effectively improve their clinical symptoms, and is suitable for clinical application. A popularization of this concept in clinical practice is worth considering, but further research and follow-up with a higher methodological quality and longer intervention time are needed to confirm its efficacy.

## 1. Introduction

Idiopathic tinnitus refers to a kind of subjective tinnitus of unknown cause in clinic, that is, no distinct abnormality is found through the current examination, or there is a lack of clear causal relationship between abnormal examination results and tinnitus [1, 2]. It not only refers to the symptoms of tinnitus but also can be used as an independent disease. The onset of idiopathic tinnitus is acute or chronic, with or without hearing and psychological disorders, which is usually associated with hearing loss, noise exposure, aging, and stress. The auditory sensitivity in tinnitus population is 40-86% [3, 4]. Most research reports show that the prevalence of adult tinnitus is about 10-19%, and in recent years, the prevalence of adult tinnitus is increasing at an annual rate of 3%, and the incidence rate increases with age. It accounts for 31.4%, and about 1/3 of the elderly suffer from tinnitus for many years. People who are male, obese, or have long-term blood pressure, blood lipids, blood sugar, psychoemotional disorders, and other related diseases, or people with a history of occupational and recreational noise exposure have a higher incidence of tinnitus [5].

Currently, the specific pathogenesis of tinnitus is not completely clear. With the development of neuroimaging, neurophysiology, neuropsychology, and so on, it is believed that tinnitus is driven by the following two mechanisms: one is the bottom-up mechanism related to hearing loss, and the other is the top-down mechanism related to insufficient noise elimination [5]. The course of tinnitus is often long, which will cause great harm to the physical and mental health of patients, and the related social and economic costs caused by its treatment are very high. Take the United States as an example, by the fiscal year 2012, the number of veterans who had received government disability pension for tinnitus alone had exceeded 970000 [6]. Since there is no standardized treatment plan at present, nonstandard and ineffective treatment can increase the cost of national health care [7]. According to relevant statistics in the United States, the annual government pension for tinnitus is more than $2.75 billion [8]. In China, there is no specific investigation in this regard, but the economic burden brought by tinnitus treatment cannot be ignored. In addition, tinnitus has a large impact on the life quality of patients, and the functional impairment caused by it mainly includes four aspects: thinking and emotion, sleep, hearing, and concentration [9, 10].

According to traditional Chinese medicine (TCM), tinnitus can be caused by exogenous and internal injuries. The pathogenesis of tinnitus can be divided into deficiency and excess, including wind-heat invasion, qi depression, inflammation of liver fire, hyperactivity of liver yang, stagnation of phlegm fire, and blood stasis. Deficiency syndrome includes deficiency of heart blood, deficiency of lung qi, weakness of spleen and stomach, deficiency of kidney essence, and loss of kidney yang [11, 12]. According to the bottom-up tinnitus mechanism, the damage of the peripheral auditory system leads to a decrease in the input signal from the cochlea to the brain, and the central auditory structure compensates the lost signal in the form of neuroplasticity. Of note, the weak cochlear signal is gradually amplified along the auditory pathway, increasing spontaneous and synchronous neural activity, which may lead to tinnitus in varying degrees. At present, with regard to the lack of specific treatment for idiopathic tinnitus, it has been found that TCM therapy such as TCM, acupuncture, moxibustion, acupoint injection, and five elements music can reduce the loudness of tinnitus and relieve the concomitant symptoms of tinnitus [13]. Acupuncture as a traditional means of TCM, based on the theory of viscera and meridians, according to the characteristics of patients' condition, acupuncture and manipulation were selected according to syndrome differentiation, which had a good effect when treating tinnitus [14]. Numerous literature studies have shown [15, 16] that acupuncture associated with nondrug interventions has better curative effect when treating idiopathic tinnitus, the therapeutic effect is better than that of rehabilitation therapy or acupuncture alone, and it has the advantages of fewer clinical adverse reactions. However, the effectiveness of TCM when treating idiopathic tinnitus has not been internationally recognized and needs to be supported by high-quality research evidence. In addition, there are large differences between different research designs, and there are many evaluation indicators. Common clinical manifestations include insomnia, anxiety, and depression, decreased concentration, and decreased speech comprehension, or other family life and work problems, and the higher the degree of tinnitus distress, the greater the likelihood of accompanying psychological, psychosomatic, and/or psychiatric comorbidities. Therefore, timely medical treatment should be recommended for such patients, and active and effective intervention should be given. Only the effectiveness of a certain literature or the improvement of a certain evaluation index is used to illustrate the clinical efficacy of TCM acupuncture associated with mind-body intervention when treating idiopathic tinnitus. The results are unconvincing and inconsistent across numerous studies. Under this background, it is very necessary to carry out further research on the efficacy of acupuncture associated with physical and mental intervention when treating idiopathic tinnitus. Therefore, this study systematically, quantitatively, and comprehensively analyzed the results of multiple independent studies of the same kind through. The purpose of this study was to evaluate the clinical efficacy of acupuncture combined with physical and mental intervention in the treatment of patients with idiopathic tinnitus through meta-analysis and to provide an objective basis for clinical application.

## 2. Research Contents and Methods

### 2.1. The Sources and Retrieval Methods of Documents

Search PubMed, EMBASE, ScienceDirect, Cochrane Library, China Journal full-text Database (CNKI), VIP full-text Database (VIP), Wanfang Database, and Chinese Biomedical Literature data (CBM); search relevant Chinese journals, conference papers, degree papers, etc.; and collect relevant data about acupuncture associated with physical and mental intervention when treating idiopathic tinnitus. Literature retrieval was carried out in the way of free words and subject words, with the key words of TCM acupuncture, physical and mental intervention, idiopathic tinnitus, tinnitus symptoms, improvement effect, meta-analysis, TCM acupuncture; idiopathic tinnitus; symptoms of tinnitus, etc., from January 2010 to March 2022.

### 2.2. Literature Inclusion and Exclusion Criteria

#### 2.2.1. Literature Inclusion Criteria

(1) Research type: all the controlled trials (CT) of acupuncture associated with physical and mental intervention when treating idiopathic tinnitus, the search languages are Chinese and English; (2) object of study: patients with idiopathic tinnitus were clearly diagnosed; diagnostic criteria of western medicine: refer to the consensus of 2012 tinnitus experts and diagnostic criteria of idiopathic tinnitus in interpretation [17]; TCM syndrome differentiation criteria: refer to the TCM diagnostic criteria of tinnitus in the Clinical Research guidelines to treat tinnitus with new drugs of TCM [18]; (3) intervention measures: the study group received physical and mental intervention measures such as acclimatization therapy/five elements music therapy/cognitive behavioral therapy/TCM horn music, while the control group only received acupuncture or simple physical and mental intervention

#### 2.2.2. Literature Exclusion Standard

(1) It is not a control study; (2) the data report is incomplete and the data cannot be used; (3) repeat the research content and take the latest research; (4) the evaluation of the curative effect of the study was not noticeable

### 2.3. Quality Evaluation and Data Extraction

1. *Bias Risk Assessment Contained in the Study*. Evaluation was performed using the bias risk assessment tool recommended in Cochrane System Review Manual 5.3
2. Data extraction and literature screening are done independently by two researchers, who collect literature, extract data, evaluate quality, and cross-check the results. When there are differences in opinion, discuss and resolve them or ask the third researcher for help. Note that Express document management software and Excel office software were used to manage and extract research data. If the data contained in the literature is incomplete, contact the author of this article to supplement it. The contents of data extraction contained (1) basic information: author, publication time, number of cases; (2) intervention measures: scheme, course of treatment; and (3) outcome indicators: total clinical effective rate, tinnitus disability assessment scale (THI) score and tinnitus evaluation questionnaire (TEQ).

### 2.4. Statistical Processing

RevMan5.3 software was adopted for meta-analysis. Counting data was indexed by relative risk (OR), and measurement data was indexed by mean difference (MD). The point estimate and 95% confidence interval (CI) of each effect are given. *χ*^2^ test was adopted for heterogeneity test, and *I*^2^ was adopted to judge the heterogeneity. Fixed effect models are used if there is no heterogeneity; if there is heterogeneity, subgroup analysis, sensitivity analysis, or descriptive analysis are used; and the random effect model is used if there is heterogeneity. The difference exhibited statistically noticeable (*P* < 0.05). Furthermore, the inverted funnel chart is drawn to measure the publication bias of the literature, and the Eggers's test is used to test the asymmetry of the funnel chart. Whenever the *P* value of this test is less than 0.1, the trim and fill method can be used to correct the funnel chart and adjust the effect of the potential release deviation.

## 3. Results and Analysis

### 3.1. The Results of Literature Retrieval and the Basic Situation of Literature Inclusion

We used a computer database to retrieve 1542 articles, 413 articles were eliminated after removing repeated studies, and 128 were retrieved by reading the titles and abstracts, after excluding irrelevant studies, reviews, case reports, and noncontrol literature, 74 articles were obtained, of which 69 had incomplete data and failed to highlight main outcomes, and finally contained 5 CT [13–20]. There were 282 samples analyzed by meta. The screening diagram of the literature is shown in Figure 1, and the basic characteristics of the contained literature are shown in Table 1.

### 3.2. Evaluation of the Quality of the Methodology Contained in the Literature

The five CT articles contained in this meta-analysis reported the baseline health status of the patients. All CT mentioned “random allocation,” but did not specify the random method, and gave detailed intervention measures and treatment course. The reasons and number of blind method and lost follow-up or withdrawal were not described in detail in 5 CT articles. According to the Jadad scale, we can see that the CT of 5 articles is less than 2 points. The risk bias analysis is shown in Figures 2 and 3.

### 3.3. Meta-Analysis Result

#### 3.3.1. Treatment Effective Rate

There were 5 CT studies contained in this study, with 282 samples. A meta-analysis was carried out on the treatment effectiveness. The results of the heterogeneity test indicated that Chi^2^ = 1.94, df = 3, *P* = 0.58, and *I*^2^ = 0%, showing that the research data contained in the study show distinct heterogeneity, and the fixed effect model was adopted to analyze (Figure 4). It is suggested that acupuncture associated with physical and mental intervention has a noticeable effect on idiopathic tinnitus.

#### 3.3.2. THI Scoring

There were 5 CT studies contained in this study, with 282 samples. The meta-analysis of THI scores after treatment was performed. The results of the heterogeneity test indicated that Chi^2^ = 22.26, df = 3, *P* < 0.0001, and *I*^2^ = 87%, showing that the research data contained in the study show distinct heterogeneity. The random effect model was adopted to analyze (Figure 5). The THI score of the study group after treatment was noticeably lower (*P* < 0.05), suggesting that acupuncture associated with physical and mental intervention is helpful for the recovery of patients with idiopathic tinnitus.

#### 3.3.3. TEQ Score

There were 5 CT studies contained in this study, with 282 samples. Meta-analysis was performed on the severity classification of tinnitus after treatment. The results of the heterogeneity test indicated that Chi^2^ = 16.81, df = 8, *P* = 0.03, and *I*^2^ = 52%, showing that the research data contained in the study show distinct heterogeneity, and the random effect model (Figure 6) analysis shows that the severity of tinnitus in the study group after treatment was noticeably lower (*P* < 0.05).

#### 3.3.4. Publication Bias Analysis

The inverted funnel chart was used to analyze the publication bias of the study with the treatment efficiency as the outcome index (Figure 7). The results indicated that most of the funnel charts were symmetrical and a few were asymmetrical, suggesting that there was a certain publication bias in the contained literature. This may be relevant to the heterogeneity of the study and the small number of contained literatures.

## 4. Analysis and Discussion

This study systematically, quantitatively, and comprehensively analyzed the results of multiple independent studies of the same kind through. Meta-analysis was performed to assess the clinical efficacy of acupuncture in the treatment of patients with idiopathic tinnitus in relation to physical and psychiatric interventions and to provide an objective basis for clinical application. With the aggravation of the aging population and the increase of environmental noise, the incidence of tinnitus is increasing year by year. According to epidemiological investigation, it is conservatively estimated that about 39 million elderly people in China suffer from tinnitus; 26 million tinnitus patients are seriously affected by tinnitus, and their life quality is seriously declining; 6.5 million patients are unable to live, work, and study normally because of tinnitus [24]. Tinnitus is still poorly understood as far as its mechanism is concerned. Some researchers such as Lee et al. [25] believe that the abnormal electrical activity of nerve fibers in the auditory conduction pathway is the basis of tinnitus, and the limbic system and autonomic nervous system are involved in the formation of tinnitus. Some researcher Qiu and Liu [26] also realized that nonauditory problems such as mental psychology, sleep, anxiety, and depression can also cause tinnitus and pointed out that after psychological and sleep problems were improved, tinnitus-related symptoms were also improved. In fact, in addition to ear surgery, diseases caused by tinnitus through surgical treatment can play a better effect, most other tinnitus can only be symptomatic treatment. Western medicine through the intervention of the primary disease, moderate improvement of inner ear microcirculation, and nutritional nerve drug treatment can improve tinnitus symptoms to a certain extent, but the cost of long-term use of western medicine is high, which will restrict patients with limited economic conditions.

The theory of TCM considers that the liver and the ear are closely related to the physiological functions, and the long-term emotional discomfort can lead to stagnation of liver qi, loss of relaxation, stagnation of qi mechanism, imbalance of ascending and descending, stagnation of fire for a long time, and stagnation of fire circulation. After disturbing the orifice, the disease will cause tinnitus. Therefore, liver-qi stagnation syndrome is a common syndrome of tinnitus. The “Nei Jing” clearly records tinnitus and expounds the pathogenesis of tinnitus from the perspective of TCM, which believes that the occurrence of tinnitus is relevant to the internal organs and is closely relevant to the liver, spleen, and kidney. Yao et al. [13] believe that most of the patients with modern tinnitus are “liver depression,” and the treatment of tinnitus from “liver depression” has received a good clinical effect. Acupuncture therapy in the external therapy of TCM shows a certain potential when treating tinnitus because of its low cost and outstanding effect. Acupuncture can improve the microcirculation of the inner ear, correct the hypoxia-ischemic state of cochlear cells, and regulate the release of neurotransmitters so as to repair inner ear cells and improve hearing. Researcher Gong et al. [27] evaluated the current situation of acupuncture treatment of tinnitus in China through meta-analysis and concluded that acupuncture therapy is distinctly better than drug therapy. This further provides a theoretical basis for acupuncture treatment of tinnitus. At present, there are many methods to treat tinnitus in western medicine, including masking therapy and acclimatization therapy, but the curative effect is unstable, so it is necessary to seek a more effective treatment of tinnitus.

The expert consensus in China pointed out that idiopathic tinnitus should be treated with tinnitus combined management (TCM), that is, tinnitus counseling, behavioral cognitive therapy, drug therapy, and sound therapy; and psychological counseling is the key (1). The American guidelines for Clinical Application of Tinnitus focus on persistent annoying tinnitus (the course of disease > 6 months). The guidelines believe that tinnitus can be improved spontaneously and lack of high-quality evidence to treat new tinnitus. It is considered to be related to the medical model of family doctors in the United States. In the United States, acute tinnitus is mainly treated by family doctors, and it is often beyond the acute stage when transferred to an ear, nose, and throat specialist for treatment. Often lose the opportunity to treat new tinnitus. This guide recommends cognitive behavioral therapy, sound therapy, hearing aid evaluation, etc. The European guidelines for multidisciplinary tinnitus: diagnosis, evaluation, and treatment strongly recommend cognitive behavioral therapy and cochlear implants for tinnitus patients with hearing loss, because the existing evidence shows that treatment measures may do more harm than good. They are opposed to repeated transcranial stimulation and drug therapy and do not comment on acclimatization therapy, sound therapy, and acupuncture therapy because of the low level of existing evidence [28, 29]. The clinical practice guide for the diagnosis and treatment of chronic tinnitus in Japan [30] discusses the treatment of chronic tinnitus (the course of disease is more than 3 months). In recent years, the therapeutic effects of tinnitus are quite different, and even the conclusions are contradictory. The German “Tinnitus Diagnosis and Treatment Outline” mainly refers to the treatment plan for sudden deafness when treating idiopathic tinnitus, but the efficacy lacks high-quality clinical evidence support.

Associated with the results of this study, there were 5 CTs contained, with 282 samples. Meta-analysis was conducted on the treatment effective rates. The results of the heterogeneity test indicated that Chi^2^ = 1.94, df = 3, *P* = 0.58, and *I*^2^ = 0%, showing that the research data contained in the study show distinct heterogeneity. The fixed effect model analysis indicated that the treatment effective rate of the study group was noticeably better (*P* < 0.05). This shows that acupuncture associated with physical and mental intervention is effective when treating idiopathic tinnitus. From the literature contained in this study, a large number of studies on acupuncture associated with physical and mental intervention when treating idiopathic tinnitus have been carried out in China, including random control group, double-blind, and multicenter high-level research. It shows that TCM acupuncture associated with physical and mental intervention has high clinical value for patients with idiopathic tinnitus. The reason why this treatment scheme has a good curative effect is that acupuncture therapy can cure both the symptoms and root causes, starting with the source of the disease and selecting acupoints. It can not only noticeably improve the inner ear microcirculation and cochlear cell ischemia and hypoxia but also repair inner ear cells, noticeably improve the hearing level of patients, and generally not easy to relapse after treatment. Physical and mental intervention can systematically improve the physical and mental state and life quality of patients and further enhance the clinical efficacy. Meta-analysis was performed on the THI score and tinnitus severity classification after treatment. The results of the heterogeneity test indicated that THI score: Chi^2^ = 22.26, df = 3, *P* < 0.0001, and *I*^2^ = 87%; severity of tinnitus: Chi^2^ = 16.81, df = 8, *P* = 0.03, and *I*^2^ = 52%; the results indicated that the research data contained in the study show distinct heterogeneity. According to the random effect model analysis, the THI score and TEQ score of the study group were noticeably lower (*P* < 0.05). It is suggested that acupuncture associated with physical and mental intervention is helpful to the recovery of patients with idiopathic tinnitus. The decrease of THI score and TEQ score also fully confirmed the science and effectiveness of this treatment scheme. Acupuncture and physical and mental intervention treatment can noticeably improve the clinical symptoms of patients and accelerate the recovery of their condition. It also shows that this treatment scheme has a broad prospect of clinical application. The same idea can be found in the study put forward by Chen et al. [31]. They have applied new methods in the study, and the conclusions drawn can also give some support to this study. This paper still have some limitations: (1) the inclusion and exclusion criteria are stricter, and the final number of contained literature is less; (2) the follow-up time of all studies is short, so there are some limitations; (3) the evaluation of quality methodology contained in the literature is not high, and there is diversity in the use of acupuncture methods, the type of control group, the selection of outcome indicators, and physical and mental intervention measures, which increases the heterogeneity among studies. More large samples and high-quality randomized controlled trials are needed to provide evidence support for the efficacy of acupuncture when treating idiopathic tinnitus; (4) this paper failed to find the source of heterogeneity through subgroup analysis, which needs to be followed up by scholars to provide more support for acupuncture associated with physical and mental intervention when treating idiopathic tinnitus, and more high-quality controlled trials need to be performed to verify it.

## 5. Conclusion

To sum up, acupuncture associated with physical and mental intervention is effective when treating idiopathic tinnitus, which can noticeably reduce the severity of tinnitus, reduce the discomfort caused by tinnitus, enhance their hearing level, and improve their life quality. This conclusion is consistent with the original literature.

## Figures and Tables

**Figure 1:** The screening diagram of the literature.

**Figure 2:** Risk of bias.

**Figure 3:** Risk of bias summary.

**Figure 4:** Forest plot of meta-analysis of effective rate of treatment.

**Figure 5:** Forest plot of meta-analysis of THI score.

**Figure 6:** Forest plot of meta-analysis of TEQ score.

**Figure 7:** Funnel chart with effective treatment.

**Table 1:** Basic characteristics of literature.

Include the literature	Year of publication	*N* (*C*/*T*)	Intervention method		Outcome index	Course of treatment	Stochastic method	Blind or not
			*C*	*T*				
Liu and Feng [19]	2017	24/24	Vinpocetine + acupuncture	Vinpocetine + acupuncture therapy + acclimatization therapy	①②	1 month	Not mentioned	No
Wang and Wang [20]	2016	27/27	Dialectical acupuncture	Dialectical acupuncture + five elements music therapy	①②	4 weeks	Not mentioned	No
Zhang et al. [21]	2021	40/40	Cognitive behavioral therapy	Acupuncture therapy + cognitive behavioral therapy	②	4 weeks	Not mentioned	No
Guan [22]	2019	20/20	Acupuncture	Acupuncture therapy + horn music of TCM	①③	84 d	Not mentioned	No
Guan and Han [23]	2021	30/30	Acupuncture	Acupuncture therapy + psychological intervention + sound therapy	①②③	28 d	Not mentioned	No

Note: *C*: control group; *T*: research group. ① Treatment effective rate; ② THI score; ③ TEQ score.

## Data Availability

The datasets used and analyzed during the current study are available from the corresponding author upon reasonable request.
